The article "The New Media Environment Presents Challenges and Opportunities for Music Education in Higher Education" was retracted in 2023. Reasons: signs of a paper mill; suspected computer-generated content; unreliable results or conclusions; lack of ethics approval or compliance.

# The New Media Environment Presents Challenges and Opportunities for Music Education in Higher Education

**DOI:** 10.1155/2022/9261521

**Published:** 2022-07-13

**Authors:** Yunzhang Xu

**Affiliations:** ^1^Taizhou University, Music Academy, Taizhou, Jiangsu 225300, China; ^2^Nanjing University of the Arts, Nanjing, Jiangsu 210013, China

## Abstract

Educational reform is essential. The revolution of multimedia technology and network technology is having a profound impact on the traditional teaching system, teaching methods, and training content. The learner-centered online learning model is rapidly developing. Research shows that, based on new media concepts and technology applications, music teaching platforms can be created and researched through limited forms of music teaching in colleges and universities and new media platforms. The survey results of the practice and role of new media in the process of assisting music teaching in colleges and universities show that most students have a positive attitude towards the new media teaching assistant method in public music courses in colleges and universities and are very interested in this method. Students' aesthetic, analytical, expressive, and collaborative abilities are also enhanced at all levels. The average score of the test class was 8.8 points higher than that of the control class, and the average score was 10.78% higher. The results show that the application of new media in college music teaching is effective.

## 1. Introduction

The book *International Vision of Chinese Music in the Context of the Internet*, edited by Yu Hui and published by Zhejiang University Press in January 2019, discusses the state and form changes of external communication of music in the Internet era against the background of the globalization process of Chinese music, which lays the foundation for the reform mode of music education in colleges and universities in China [1, 2]. As the main position for training music teachers of basic education in the new era, ordinary colleges and universities must build a professional core curriculum group system that meets the needs of basic education in the new era, the requirements of aesthetic education, and the standard of normal professional certification.

Figure 1 shows the implementation process of teachers' application of new media to assist teaching. In addition, the learning styles and learning needs of students in the information environment are also changing, which is very different from the previous generation. Therefore, in order to improve the quality of college music education and support its reform and reform, it is necessary to study the introduction and use of new media in college music education [3].

The article "The New Media Environment Presents Challenges and Opportunities for Music Education in Higher Education" was retracted in 2023. Reasons: signs of a paper mill; suspected computer-generated content; unreliable results or conclusions; lack of ethics approval or compliance.

## 2. Literature Review

The first is to introduce the talent training mode of music education specialty and analyze the talent training mode, such as music teacher education, a TA liberal arts college, and multivariate analysis of degree persistence of undergraduate music education majors. Second comes the impact of education related policies on music education, such as reflections on educational policy reforms and education. The third is the influence of multiple factors on music education, such as socialization of underground music education major in professional development partnership model, connect in gifts to practice: the development of an underground student's philosophy of music education. The fourth is the analysis and research on the cooperation between music education major and other majors; for example, coordination is the key: a report of a joint project of music education and elementary education majors, and so on.

This paper studies and analyzes the courses offered by the major of music education in colleges and universities, including the reform of the curriculum of music education, the application of new technology in the curriculum of music education, and the teaching thinking on skills of the major of music education in colleges and universities; for example, Wen, and others said that “the Ministry of education has also promulgated the music curriculum standard for full-time compulsory education (experimental draft), which puts forward requirements for self-playing and self-singing ... How to do well in self-playing and self-singing and let students master professional self-playing and self-singing skills has become the focus of research in colleges and universities [4].” Bălilescu et al.'s study of the so-called flip classroom mainly will adjust inside and outside class time students to learn at their own discretion is a kind of can cultivate students' autonomous learning consciousness and ability of independent exploring new education pattern, the education mode based on the information platform for education or education software [5]. Lai et al.'s research suggests that, in the actual process of music teaching in, should be performed according to the teaching content of different grades of data collection, and the difference should have depth and the difficulty of theory of cross-cutting, cannot machine-made, grade, school level, and so on, should be based on students scientifically for the choice of teaching content and design [6]. Guo et al. believe that due to the backward technology and equipment and unsatisfactory teaching feedback of traditional audio-visual training courses, students are less interested in learning such knowledge. In order to make students face up to this course, teachers can use some information software to assist teaching in the process of music teaching [7].

The article "The New Media Environment Presents Challenges and Opportunities for Music Education in Higher Education" was retracted in 2023. Reasons: signs of a paper mill; suspected computer-generated content; unreliable results or conclusions; lack of ethics approval or compliance.

Carry out macro analysis and research from the talent training mode of music education major in colleges and universities; for example, Han et al. mentioned in the article that “the current situation and social needs of talent training of music education majors in colleges and universities force the renewal and upgrading of teaching methods, contents and curriculum of music education majors, and the proposal of core literacy provides guidance for the improvement and long-term development of students majoring in music education in colleges and universities ... From focusing on simple professional knowledge teaching to more comprehensive application-oriented talent training” [8]. Onwubiko and Calilhanna found that the professional core curriculum is the main carrier of cultivating the core literacy of students majoring in music education. The future role of music education major students in the new era is music teachers of basic education, whose core literacy includes four dimensions of “disciplinary literacy, interdisciplinary literacy, teacher ethics literacy, and introspection literacy” [9]. Li constructed professional core curriculum group by centering on “professional ability” and “teaching ability” in “discipline accomplishment” and taking “playing, singing, dancing, and editing teaching” as the standard for music education major students [10]. Nazmine et al. in their research found that the discipline literacy was as follows: the ability to play one or two commonly used instrumental music in China and the West; the ability to improvise piano accompaniment in music textbooks for primary and secondary schools; the ability to play and sing songs by themselves; the ability to play and see piano; and so on. The core ability of playing is the ability to play piano [11].

On the basis of existing research, combined with the analysis of the current situation of public music education in the new media environment, the opportunities and challenges faced by music education in colleges and universities under the influence of music education are analyzed. *New Media*. The survey results show that most students have a positive attitude towards the new media teaching assistant method in public music classes in colleges and universities and are very interested in this method. Students' aesthetic, analytical, expressive, and collaborative abilities are also enhanced at all levels. The average score of the test class was 8.8 points higher than that of the control class, and the average score was 10.78% higher. The results show that the application of new media in college music teaching is effective.

The article "The New Media Environment Presents Challenges and Opportunities for Music Education in Higher Education" was retracted in 2023. Reasons: signs of a paper mill; suspected computer-generated content; unreliable results or conclusions; lack of ethics approval or compliance.

## 3. Research Methods

### 3.1. Investigation and Analysis on the Current Situation of Public Music Teaching

From the teaching effect and students' feedback in recent years, students have great interest in the course, but because there are only two class hours per week, the amount of information taught and presented by teachers in the classroom often cannot meet the needs of students. The survey was conducted in May 2021 with the assistance of the instructor. The students completed the questionnaire and took it back on the spot. A total of 186 questionnaires were distributed, 186 were recovered, and 182 were valid, with an effective rate of 98.38%. Therefore, the results of the questionnaire survey are valid. In order to save time, 50 samples were randomly selected according to the proportion of the number of people in each class (32 ^*∗*^ 50/182 = 8 in the class of information management, 51 ^*∗*^ 50/182 = 14 in the class of modern educational technology, 51 ^*∗*^ 50/182 = 14 in the class of English Education (1), 52 ^*∗*^ 50/182 = 14 in the class of English Education (2), and 52 ^*∗*^ 50/182 = 14 in the class of English Education (2)). The analysis methods and results are described in Tables 1–9 below.

It can be seen from Table 1 that the teaching conditions and environment of the school can fully meet the teaching needs of public music courses in colleges and universities.

According to the statistical results, students believe that in the teaching and learning of this course, the existing problems are that firstly, there is not enough time for communication between teachers and students, and then students are still in a passive learning state, too dependent on teachers, and lack of awareness of knowledge management after class. Teachers have not given full play to the advantages of network in teaching, and students do not have time to reflect or internalize knowledge. Therefore, in view of the above problems, teachers must adopt corresponding strategies and Reform in future teaching.

The results show that students hope that the forms of teachers' teaching can become diversified, and most students are willing to participate in learning activities.

The statistical results show that students hope to be exposed to more music tracks as much as possible through the study of this course, and nearly half of the students want to have an in-depth understanding of famous music and hope to be widely involved. It can be seen that most students are eager to master more music knowledge.

The statistical results show that more than half of the students' music feeling ability is low, and the students' music literacy needs to be further strengthened.

The article "The New Media Environment Presents Challenges and Opportunities for Music Education in Higher Education" was retracted in 2023. Reasons: signs of a paper mill; suspected computer-generated content; unreliable results or conclusions; lack of ethics approval or compliance.

The statistical results show that the study of music class can first cultivate sentiment and then broaden the scope of knowledge, adjust the tense study life, and change the way of learning. Generally speaking, the purpose of students' learning music is to improve their own quality and self-cultivation.

The reason is that in the conventional music education and teaching in colleges and universities, although students are more interested in music courses, due to the poor foundation of students, many students only stay in the love and understanding of popular singers and pop music and lack enthusiasm and understanding of traditional Chinese folk music and classical Western classical music. Students' learning style is mainly “passive acceptance.” There is little communication between teachers and students, and there is a lack of mutual cooperation between students. Students' learning enthusiasm is not high, and their learning methods are single. In addition to listening in class, there are no practical activities of active learning after class. Most students' mastery of music and cultural knowledge is limited to the information transmitted by classroom teachers. The scope of knowledge is narrow, and even some students forget it after listening to it.

### 3.2. Connotation and Characteristics of Music Education in Colleges and Universities under New Media

#### 3.2.1. Connotation

Music education refers to the educational activity that changes the aesthetic consciousness, cultivates the sentiment, develops the thinking ability, and makes the educatee become a fully developed member of the society by imparting music knowledge and skills to the educatee. As a national base for cultivating high-quality talents, colleges and universities bear important responsibilities. As an important part of the higher education system, music education plays a very important role in cultivating the overall quality and all-round development of contemporary college students. Like art colleges and universities, ordinary colleges and universities offer music courses for art education. The teaching object of music education in colleges and universities should refer to the majority of students who are not art majors. The purpose of music education in colleges and universities is to cultivate all-round developed talents, improve college students' aesthetic ability and artistic appreciation through music edification, develop thinking ability and creativity, and carry out school music education in an organized, planned, and purposeful way [12].

Music education, as one of the important categories of educational content, also follows the wave of new media, which has brought earthshaking changes to the traditional music teaching mode. Music education in the new media era is a new teaching model formed by integrating new media technology and music education and integrating the characteristics of music art and the concept of music personalized education. The education model is not constrained by time and space and provides high-quality music sharing resources.

The article "The New Media Environment Presents Challenges and Opportunities for Music Education in Higher Education" was retracted in 2023. Reasons: signs of a paper mill; suspected computer-generated content; unreliable results or conclusions; lack of ethics approval or compliance.

#### 3.2.2. Features

*(1) Openness*. Under the traditional education mode, the music education industry is relatively closed, and some music learning resources, including music scores, records, musical instruments, music works, and audio and video materials of performing artists, are only open to music majors. With the rapid development of new media, a variety of music teaching resources, including music scores, artist performance videos, and publications, can be easily searched and obtained online. Therefore, new media has become the communication channel of digital music resources. These network platforms are not only cost-effective, but also provide free resource sharing. Music under the new media makes it easier to obtain various learning resources. This new educational model subverts the traditional music education and promotes the rapid sharing of music activities [13]. In addition to openness, music learning resources can be shared through online teaching. For example, many colleges and universities let their excellent music teachers choose the teaching contents loved by students and record open classes and put them on the learning platform. Not only for their students, but also for other different types of college students so as to realize the sharing of high-quality teacher resources. In addition, the online teaching mode is not affected by geographical factors. Colleges and universities in remote areas can also obtain the same educational resources, teachers, and teaching contents as those in developed areas. For areas with backward educational resources, it broadens students' vision and realizes educational fairness to a certain extent.

*(2) Timeliness*. Students can watch the important and difficult points and difficult knowledge taught by teachers in time after class and can watch and review at any time, which is not easy to forget. It is one of the biggest advantages of online music education mode. In addition, as a means of transmitting information and obtaining data, new media makes the emergence, dissemination, and reception of music and other music activities timelier. At present, major music websites and learning resource libraries are gathered in the new media, and a large number of music app software in the mobile terminal are also launched. NetEase Cloud, QQ Music, and other software have attracted hundreds of millions of users. Most of the users are college students, which is convenient for them to accept and enjoy music anytime and anywhere. In terms of music creation and dissemination, music creators can create a complete song online through digital technology, and the music works will be immediately transmitted to users' hands after being released.

*(3) Initiative*. With the continuous advancement of educational reform, we pay more attention to the student-centered teaching concept and highlight the dominant position of students in teaching activities. Learning in the Internet plus education era emphasizes learners' initiative. College students should have self-control and be able to find the content they are interested in in a large number of learning resources, which is no longer the state of teachers “chasing after learning” and “catching up with learning.” The music learning mode in the new media era should be that learners take the initiative to obtain and use the information platform with the help of the network platform, choose the music learning content and teachers they are interested in, choose their own learning methods, study independently, dare to distribute learning results on the learning platform, share learning experience with others, and improve learning quality through autonomous learning ability.

The article "The New Media Environment Presents Challenges and Opportunities for Music Education in Higher Education" was retracted in 2023. Reasons: signs of a paper mill; suspected computer-generated content; unreliable results or conclusions; lack of ethics approval or compliance.

### 3.3. New Media-Based Learning

The teaching process based on new media is a process in which learners publish their learning experiences and materials online in the form of logs or videos on the learning platform, strengthen the management of students' learning process, expand the scope of students' access to knowledge, enhance the communication between teachers and students as well as students and students, improve students' learning interest, and improve students' learning effect [14].

Design of several stages of experimental research on the application of new media in music education and teaching in Colleges and universities is as follows.

#### 3.3.1. Preparation Stage

After the establishment of the music education platform, 42 people in the professional class of modern educational technology were selected for publicity and demonstration operation, and the whole class was allowed to try it on the Internet to make timely adjustments in case of problems.

#### 3.3.2. Application Stage

After the preliminary preparation, the teaching publicity and formal experiment based on the learning platform were carried out in the professional class of modern educational technology, and the comparative teaching under the conventional teaching mode was carried out in the professional class of computer information management in our college [15].

The article "The New Media Environment Presents Challenges and Opportunities for Music Education in Higher Education" was retracted in 2023. Reasons: signs of a paper mill; suspected computer-generated content; unreliable results or conclusions; lack of ethics approval or compliance.

#### 3.3.3. Analysis and Summary Stage

The final comprehensive test is conducted for each class, and the questionnaire survey is conducted for the experimental class. Combined with the comprehensive learning performance of the two classes, the analysis and summary of public music teaching in colleges and universities based on the new media learning platform is made [16, 17]. In the experiment of applying new media assisted instruction, several processes are designed, such as goal analysis task definition, using the platform to provide information resources, organization, guidance, helping students' collaborative learning summary, and guiding and evaluating students' learning.

## 4. Result Analysis

### 4.1. Carrying Out Experiments and Experimental Results

The experimental teaching research has been carried out since June 2021, and a questionnaire survey has been conducted on the students in the experimental class at the end of the term. The subjects of the survey were 42 students in the experimental class of modern educational technology major in our school. A total of 42 questionnaires were distributed, 42 were recovered, and 42 were valid.

The data in Tables 10–20 below are all from the questionnaire of 42 students.

Statistics show that nearly two-thirds of students have their own computers.

The statistical results show that most students can use computers connected to campus network or the Internet after class. Each student dormitory has 5–8 computers bought by students. The school has campus Internet cafes. Students can basically use computers conveniently.

The statistical results show that some students think it is important to communicate and discuss with their classmates, while only students think it is not important. This shows that communication is necessary in learning, so we should create a space for students to communicate, stimulate students' consciousness and enthusiasm in learning, and make students change from passive acceptance of knowledge to active exploration of knowledge.

The statistical results show that all students can log in to the new media music teaching blog according to the requirements of teachers.

The statistical results show that most students log in to the music teaching platform more than 10 times a month. Some students log in almost every day, and only some students log in less than once a week. This shows that the network is not strange to students. It is a modern information tool that students like.

The statistical results show that most students log in to the music teaching platform for a long time each time, indicating that students are more interested in it.

The article "The New Media Environment Presents Challenges and Opportunities for Music Education in Higher Education" was retracted in 2023. Reasons: signs of a paper mill; suspected computer-generated content; unreliable results or conclusions; lack of ethics approval or compliance.

The statistical results show that the main reason for students to log in to the music education platform is to view useful learning information, then communicate with teachers and students to understand the learning status of other students, teachers' requirements, hobbies, or habits, and finally to relax the tense learning life.

The statistical results show that most students are most willing to check useful learning information and expand their music vision after logging in to teacher Xie's music teaching blog network.

For the application of music teaching platform for auxiliary teaching, the results of which aspects of students' abilities have been improved are shown in Figure 2 below. The statistical results show that more than 90% of the students believe that their aesthetic ability has been improved, and most of the students also believe that their cooperation ability, autonomous learning ability, and lifelong learning ability have been improved at the same time. On the other hand, it reflects that most of the students are not aware of the change of their own innovation ability.

### 4.2. Comparative Analysis

The pretest of the basic music knowledge of the experimental class and the control class was carried out. After one semester of the experiment, the posttest of the basic music knowledge of the experimental class and the control class was carried out again in the same month. For the comparative analysis of the two test results, see Tables 21 and 22. We try to find out how this way of learning through the application of new media music teaching platform can help students learn public music courses in colleges and universities.

Since the number of people in the two different populations in this experiment is larger than that in the other two populations, which belongs to a large sample, *Z*-test is used to statistically analyze the results to test whether the overall differences represented by them are significant [18, 19].

*Z*-Test is a common method of hypothesis test, and the hypothesis test of overall proportional parameters is a common hypothesis test problem, which is described in detail in the applied statistics textbook. There are usually two methods to test the proportional parameter *p*: one is the accurate test of small samples; the other is large sample approximation test. Without losing generality, take the right test as an example, set:

(1) $$\begin{array}{c} h_{0}:p\leq p_{0}, \end{array}$$

(2) $$\begin{array}{c} h_{1}:p>p_{1}. \end{array}$$

The test under small samples is based on binomial distribution *B* (*n*, *P*), with

(3) $$\begin{array}{c} P\left(\text{Refused to }h_{0}|h_{0}\right)=P\left(X\geq c,X-B\left(n,p_{0}\right)\right). \end{array}$$

When the sample size is large, according to the central limit theorem (De Moivre–Laplace theorem), $\hat{p}$ approximately obeys the normal distribution:

(4) $$\begin{array}{c} \hat{p}-N\left(P,\frac{P\left(1-p\right)}{n}\right). \end{array}$$

Then, there are the following test statistics:

(5) $$\begin{array}{c} z=\frac{\hat{p}-p_{0}}{\sqrt{p_{0}\left(1-p_{0}\right)/n}}. \end{array}$$

Z∼*n* (0,1), formula (1) is the form of *Z*-test statistics commonly used in textbooks.

The article "The New Media Environment Presents Challenges and Opportunities for Music Education in Higher Education" was retracted in 2023. Reasons: signs of a paper mill; suspected computer-generated content; unreliable results or conclusions; lack of ethics approval or compliance.

However, the author often finds in teaching practice that some students often replace the denominator *p*_0_ in the statistics of formula (5) with *p* and replace the *Z*-test with *t*-test, as shown in the following formula.

(6) $$\begin{array}{c} T=\frac{\hat{p}-p_{0}}{\sqrt{\hat{p}\left(1-\hat{p}\right)/n}}. \end{array}$$

The test of the overall mean value is still the traceability test. If a random variable *x* is only a normal random variable, two tests can be used for the test of *E* (*x*) = *U*. One is the *Z*-test with known variance, and the test statistic is formula (7); the other is the *t*-test with unknown variance, and the test statistic is expressed in equation (8).

(7) $$\begin{array}{c} Z=\frac{\bar{X}-u_{0}}{\sigma /\sqrt{n}}, \end{array}$$

(8) $$\begin{array}{c} T=\frac{\bar{X}-u_{0}}{S/\sqrt{n}}. \end{array}$$

When *x* obeys the (1–0) distribution with parameter *P*, *N* random samples

(9) $$\begin{array}{c} \bar{X}-N\left(p,p\left(1-p\right)\right). \end{array}$$

When *n*⟶*∞*, $\bar{X}$ is the unbiased consistent estimator of *p*. Therefore, equations (7) and (8) can be transformed into equations (5) and (6), respectively.

If we broaden the horizon, we know that hypothesis testing and interval estimation are a pair of dual problems. For unknown parameters, using sample information to estimate the true value of parameters can use interval estimation, while the same sample and the same statistic can be transformed into the test of unknown parameters. In general textbooks, it is given that in the case of large samples, when the overall variance is unknown, the interval estimation of the mean is in the form of formula (7); that is,

(10) $$\begin{array}{c} \bar{X}\pm t_{a/2,n-1}\frac{S}{\sqrt{n}}. \end{array}$$

When *n*⟶*∞*, the normal approximation can also be used directly; that is,

(11) $$\begin{array}{c} \bar{X}\pm z_{a/2}\frac{S}{\sqrt{n}}. \end{array}$$

For the interval estimation of the overall proportion, replace the text with *p* and replace *s* with

(12) $$\begin{array}{c} \sqrt{\hat{p}\left(1-\hat{p}\right)}. \end{array}$$

Obviously, the use of *p*-estimated variance in interval estimation statistics still has reason to be used in the statistics used in hypothesis test. The problem encountered by the author in teaching practice is likely to be that students directly use the statistics used in interval estimation for hypothesis test analysis.

The article "The New Media Environment Presents Challenges and Opportunities for Music Education in Higher Education" was retracted in 2023. Reasons: signs of a paper mill; suspected computer-generated content; unreliable results or conclusions; lack of ethics approval or compliance.

The potential of hypothesis test is defined as follows: when *h*_0_ is false, the probability of rejecting *h*_0_, that is, 1 − *β*, the probability of not making class II errors. The purpose of potential analysis is to study the relationship between sample size, significance level, overall effect size (ES), and statistical potential. The purpose of introducing potential analysis is to compare the efficiency difference between the two test methods. Therefore, the focus of the investigation is how the potential difference between the two methods is when the sample size, significance level, and ES change. Here, the right test is still taken as an example. If the significance level is *α*, the potential function of *Z*-test is:

(13) $$\begin{array}{c} {\text{power}}_{z}=P\left(\text{Refused to }h_{0}|h_{0}\text{Is false}\right),\\ P\left(\text{Refused to }h_{0}|h_{0}\text{ Is false}\right)=p_{h_{1}}\left(\frac{\hat{p}-p_{0}}{p_{0}\left(1-p_{0}\right)/n}>z\right),\\ p_{h_{1}}\left(\frac{\hat{p}-p_{0}}{p_{0}\left(1-p_{0}\right)/n}>z\right)=1-\varphi \left(\frac{p_{0}-p+\sqrt{p_{0}\left(1-p_{0}\right)/n}}{\sqrt{p\left(1-p\right)/n}}\right), \end{array}$$

where *φ* is the normal distribution function. The potential function of *t*-test is

(14) $$\begin{array}{c} P\left(\text{Refused to }h_{0}|h_{0}\text{ Is false}\right)=p_{h_{1}}\left(\frac{\hat{p}-p_{0}}{\hat{p}\left(1-\hat{p}\right)/n}>t_{a}\left(n-1\right)\right),\\ p_{h_{1}}\left(\frac{\hat{p}-p_{0}}{\hat{p}\left(1-\hat{p}\right)/n}>t_{a}\left(n-1\right)\right)=1-T_{n-1,\lambda }\left(t_{a}\left(n-1\right)\right),\\ \lambda =\frac{p-p_{0}}{\sqrt{p\left(1-p\right)/n}}, \end{array}$$

where *t* is a noncentral *T*_*n*−1,*λ*_ distribution function whose degree is equal to *n*−1 and the noncentral parameter is *λ*.

The final examination result of the experimental class is 8.8 points higher than the average score of the control class, the pass rate is 10.78% higher, and the excellent rate is 13.54% higher.

It can be seen from the above data that before the experiment, the scores of the two classes are very close, indicating that the knowledge preparation of the two classes is very close, and there is no significant difference. After the experiment, the scores of the two classes are very significant, which proves that the form of auxiliary teaching using music teaching platform in public music courses in colleges and universities can meet the teaching requirements. On the other hand, the standard deviation of the experimental class is 7.129, which is smaller than the standard deviation of the control class is 11.135. The experimental results also show that the application of new media music teaching platform in college public music courses is more conducive to the balanced development of all students.

The article "The New Media Environment Presents Challenges and Opportunities for Music Education in Higher Education" was retracted in 2023. Reasons: signs of a paper mill; suspected computer-generated content; unreliable results or conclusions; lack of ethics approval or compliance.

### 4.3. Opportunities and Challenges in Music Education in Colleges and Universities under the New Media Environment

College music education in the new media era is mainly based on the online teaching mode. Therefore, taking the online teaching mode of college music as an example, this paper discusses the opportunities and challenges in college music education in the new media era [20].

#### 4.3.1. Opportunities

*(1) Break Through Time and Space Constraints and Reduce Teaching Costs*. Compared with traditional offline classes, online teaching has many insurmountable advantages. Relying on the Internet platform, teachers and students break through the limitation of time and space. Teachers realize synchronous teaching through live classes and asynchronous teaching through video classes. With the help of a computer and a mobile phone, students can realize their desire to study anytime and anywhere. In addition, the information-based teaching platform also provides pause, speed doubling, and playback functions, which can help students who do not understand or are distracted in class to look back repeatedly after class [21, 22].

*(2) Rich Learning Resources to Stimulate Students' Interest*. Compared with other disciplines, music education is often more relaxed and pleasant for college students, but it is often boring in the mastery of music theory and repeated practice of musical instruments. Online music teaching often covers a large number of videos and pictures, which greatly stimulate students' interest in learning. College students in the Internet era have long been inseparable from smartphones and various application software. Therefore, the online teaching mode is in line with their learning style and pace of life. A large number of musical instrument simulator apps have been developed in large quantities. Combined with big data, virtual reality (VR), artificial intelligence (AI), and other technologies, they have gathered music materials to simulate all musical instruments, breaking the traditional offline class that must rely on physical musical instruments, which not only saves costs for students, but also makes students more immersive and enhance the learning atmosphere [23, 24].

*(3) Share High-Quality Resources and Realize Cultural Exchanges*. During the epidemic, more than 24000 online courses were opened free of charge. Online learning platforms such as Moke and Superstar Teacher link maximize resource sharing [25]. Students can choose free learning resources according to their interests, and paid resources also have the function of free trial so as to truly achieve personalized education. Mu class platform spans the limitations of different regions and different learning, breaks through the traditional classroom, which only serves dozens to hundreds of people in one class, and makes the beneficiary students popularize in schools in all regions. In addition, music lovers from all over the world with different cultural backgrounds and different life experiences conduct cultural collision and exchange through online learning forums to help students with music talents so that they can carry out personalized learning and long-term learning. Therefore, online music education can stimulate students' potential and enable them to realize their own life value in music learning, in order to realize lifelong music education.

The article "The New Media Environment Presents Challenges and Opportunities for Music Education in Higher Education" was retracted in 2023. Reasons: signs of a paper mill; suspected computer-generated content; unreliable results or conclusions; lack of ethics approval or compliance.

#### 4.3.2. Challenges

*(1) Students Lack Self-Control and Poor Learning Atmosphere*. Due to the online music teaching form of “facing each other across the screen,” teachers cannot see whether students are really listening or not and cannot see the real student state of students. The student union is polarized due to different self-control. Students with strong self-control will be more strict with themselves, and students with weak self-control may go downhill.

*(2) Teachers' Teaching Methods Are Backward and Their Information Literacy Is Not High*. In addition to preparing lessons as usual, teachers should also learn to use various live broadcasting tools and teaching platforms. In college music teaching, some teachers believe that online teaching only “carries” the classroom to the network, follows the traditional teaching methods, and does not carry out personalized teaching according to the individual differences of students. This makes students gradually lose interest in learning music, and it is difficult to achieve good teaching results. Some teachers have low acceptance of information-based teaching and are unwilling to use new learning resources. They just teach in the traditional way. Students will soon feel boring and cannot concentrate on learning for a long time. Some music teachers have not systematically conducted online education and training and are not comfortable with the use of audio editing software and instrument simulator app, which also brings difficulties to the normal development of online teaching.

*(3) Due to The Limitations of Network Technology and Intelligent Terminal, The Quality of Teaching Has Decreased*. Online teaching is also affected by many external factors of force majeure. Compared with other courses, music courses have relatively high requirements for recording equipment and network connection. Subject to the instability of online teaching platform, it is easy to have a negative impact on teaching, such as asynchronous sound and picture, distorted sound effect, blurred pixels, and so on. After music is transmitted through the media, the sound quality is far lower than that of traditional classroom teaching. Students cannot really feel the real meaning that teachers want to convey and cannot reach artistic resonance so as to reduce the quality of teaching.

The article "The New Media Environment Presents Challenges and Opportunities for Music Education in Higher Education" was retracted in 2023. Reasons: signs of a paper mill; suspected computer-generated content; unreliable results or conclusions; lack of ethics approval or compliance.

## 5. Conclusion

After the experiment of new media technology-assisted teaching, through the analysis of questionnaire survey, classroom observation, conversation with students, and the results of final examination, it is concluded that the main advantages of applying it to music-assisted teaching in colleges and universities are as follows:

1. It expands students' access to music information and improves students' comprehensive quality.
2. It has changed the original learning style and stimulated the enthusiasm of students to actively participate in learning.
3. It strengthens the communication between teachers and students and students and improves students' cooperation and team awareness.
4. It is proved that the application of new media technology in music-assisted teaching in Colleges and universities is an effective tool for learning.

Generally speaking, it is applied in music education in colleges and universities. Auxiliary teaching provides a platform for teacher-student communication, resource sharing, and students' cooperative learning, breaks the restrictions of time and space, promotes students' autonomous learning, strengthens the communication between teachers and students, stimulates students' learning interest and initiative, and improves students' knowledge level and music literacy. Students' cooperation and team consciousness have also been greatly improved, which better achieves the purpose of music education in colleges and universities as improving the comprehensive quality of college students in college education.

## Figures and Tables

**Figure 1:** Implementation of teachers' application of new media assisted instruction.

**Figure 2:** Improvement of other abilities after learning on the music teaching platform.

**Table 1:** Places where teachers teach public music courses in colleges and universities.

Public music course learning places in colleges and universities	Number of people	Proportion (%)
Ordinary classroom	0	0
Multimedia classroom	50	100

The article "The New Media Environment Presents Challenges and Opportunities for Music Education in Higher Education" was retracted in 2023. Reasons: signs of a paper mill; suspected computer-generated content; unreliable results or conclusions; lack of ethics approval or compliance.

**Table 2:** Whether students are interested in the course of college public music they have studied.

	Very interested	Be interested	Uninterested	Very uninterested	Score rate *F*1
	+2	+1	−1	−2	
Number of people	14	30	5	1	0.51

From *F*1 = 0.510 > 0.5, it can be seen that students are generally interested in the course of public music in colleges and universities.

**Table 3:** Can the study time of two class hours a week meet your learning needs of this course?.

	Yes	No	No	Scoring rate *F*2
	+1	0	−1	
Number of people	12	7	31	−0.19

From *F*2 = −0.19 < 0, it can be seen that the vast majority of students believe that two class hours are far from meeting their learning needs for the course.

**Table 4:** What problems do you think still exist in the teaching and learning of this course?.

Factor	First place	Second place	Third place	Fourth place	Fifth place	Ranking index *w*_*i*_
	5	4	3	2	1	
Despite the use of multimedia teaching, teachers are still in a dominant position and students are still in a passive state of learning	18	9	10	8	5	0.236

There is not enough time for communication between teachers and students	15	17	9	6	3	0.247

The dependence on teachers is too strong, and there is a lack of awareness of knowledge management after class	4	12	17	9	8	0.195

Teachers' teaching technology and teaching means are relatively backward, and they have not given full play to the advantages of the network	8	6	7	16	13	0.175

There is no time to reflect or internalize knowledge	5	5	7	13	20	0.148

**Table 5:** What kind of music appreciation class do you like?.

	Focus on explanation	Focus on listening	Guide students to actively participate in the discussion
Number of people	9	13	28
Percentage	18%	26%	56%

**Table 6:** Your requirements for the number of tracks in the limited time of music appreciation class.

	Analyze the famous music in detail so as to master the method of appreciating famous music and seek perfection	Brief explanation of famous music so as to save time, contact more tracks, and widely read	Give consideration to both
Number of people	9	20	21

Percentage	18%	40%	42%

**Table 7:** What do you think of music appreciation teaching?.

	Combined with video appreciation, the effect is better	Music is the art of hearing	Indifferent
Number of people	29	16	5
Percentage	58%	32%	10%

**Table 8:** What benefits do you think music lessons can bring you?.

Factor	First place	Second place	Third place	Fourth place	Ranking index *w*_*i*_
	4	3	2	1	
Broaden the scope of knowledge	14	17	8	11	0.268
Cultivate sentiment, delight, and elegance	23	18	6	3	0.322
Adjust the tense study life	7	7	20	16	0.21
Changed the way of learning	6	8	16	20	0.2

The article "The New Media Environment Presents Challenges and Opportunities for Music Education in Higher Education" was retracted in 2023. Reasons: signs of a paper mill; suspected computer-generated content; unreliable results or conclusions; lack of ethics approval or compliance.

**Table 9:** Your satisfaction with public music classes.

	Very satisfied	Satisfied	Basically satisfied	Dissatisfied	Very dissatisfied
Number of people	3	7	16	23	1
Percentage	6%	14%	32%	46%	2%

**Table 10:** Do you have your own computer in school?.

	Yes	No
Number of people	27	15
Percentage	64.29%	35.71%

**Table 11:** Can you easily use the computer connected to campus network or the Internet after class?.

	Yes	No
Number of people	40	2
Percentage	95.24%	4.76%

**Table 12:** Is it important to communicate and discuss with students?.

	Important	Unclear	Unimportant
Number of people	36	5	1
Percentage	85.71%	11.90%	2.38%

**Table 13:** Have you logged in to the music teaching platform?.

	Yes	No
Number of people	42	0
Percentage	100%	0%

**Table 14:** Monthly frequency of landing on music teaching platform.

	More than 20 times	15–20 times	10–15 times	5–10 times	Less than 5 times
Number of people	4	7	13	17	1

Percentage	9.52%	16.67%	30.95%	40.48%	2.38%

**Table 15:** Time of each landing on music teaching platform.

	More than 1 hour	0.5–1 hour	15–30 minutes	5–15 (minutes)	Less than 5 (minutes)
Number of people	12	19	8	3	0

Percentage	28.57%	45.24%	19.05%	7.14%	0.00%

**Table 16:** Reasons for landing on music teaching platform (multiple choices).

	Teacher's requirements	View useful learning information	Communicate with teachers and students to understand the learning status of other students	Relax tense study life	Hobbies or habits
Number of people	24	35	31	14	16

Percentage	56.99%	83.87%	73.12%	33.33%	38.71%

**Table 17:** What are you willing to do after landing on the music teaching platform?.

	View useful learning information and expand your music vision	Exchange learning experience	Ask learning questions	Finish one's homework
Number of people	37	23	14	29

Percentage	88.10%	54.76%	33.33%	69.05%

**Table 18:** Is it agreed that the application of music teaching platform in the teaching of public art courses can assist learning?.

	Strongly agree	Basically agree	Disagree	Strongly disagree	Scoring rate *F*1
	+2	+1	−1	−2	
Number of people	22	17	3	0	0.690

From *F*1 = 0.690 > 0.5, it can be seen that students generally agree that the application of music teaching platform in the teaching of public art courses is helpful for auxiliary learning.

**Table 19:** Whether the music teaching platform has improved compared with traditional classroom teaching.

	Greatly improved	A little improved	Uncertain	Not improved	Down	Scoring rate *F*2
	+2	+1	0	−1	−2	
Number of people	18	15	7	2	0	0.583

From *F*2 > 0.5, it can be seen that students generally hold a positive attitude towards the application of music teaching platform in public music courses, which has greatly improved their music knowledge compared with traditional classroom teaching.

The article "The New Media Environment Presents Challenges and Opportunities for Music Education in Higher Education" was retracted in 2023. Reasons: signs of a paper mill; suspected computer-generated content; unreliable results or conclusions; lack of ethics approval or compliance.

**Table 20:** Teaching effect of music teaching platform.

	Very good	Good	Indifferent	Not good	Very bad	Scoring rate *F*3
	+2	+1	0	−1	−2	
Number of people	10	22	5	4	1	0.429

From *F*3 > 0, it can be seen that students have a good teaching method of using music teaching platform in public music courses.

**Table 21:** Pretest data and statistical feature analysis of experimental class and control class (pretest).

		Number of people	Average score	Standard deviation	Corresponding quadrant	Statistical characteristics
Pretest	Experimental class	42	36.07	11.177	Beta quadrant	The average level is low but scattered, and there are high-score students
	Control class	38	36.32	11.526	Beta quadrant	The average level is low but scattered, and there are high-score students

Pretest *Z* = −0.070, |*Z*| < 1.96, so there was no significant difference between the two groups.

**Table 22:** Pretest data and statistical characteristic analysis of experimental class and control class (posttest).

		Number of people	Average score	Standard deviation	Corresponding quadrant	Statistical characteristics
Posttest	Experimental class	42	78.43	7.129	Delta quadrant	The average level is high but relatively concentrated, which is in an excellent state
	Control class	38	66.74	11.135	First quadrant	The average level is low, but the degree of separation is large, and there is low meristematic

Posttest *Z* = 4.022 > 2.58, so the difference between the two groups is very significant.

## Data Availability

The labeled data set used to support the findings of this study is available from the corresponding author upon request.
